# Deep Learning for Autism Diagnosis and Facial Analysis in Children

**DOI:** 10.3389/fncom.2021.789998

**Published:** 2022-01-20

**Authors:** Mohammad-Parsa Hosseini, Madison Beary, Alex Hadsell, Ryan Messersmith, Hamid Soltanian-Zadeh

**Affiliations:** ^1^Department of Bioengineering, Santa Clara University, Santa Clara, CA, United States; ^2^AI Research, San Jose, CA, United States; ^3^CIPCE, School of Electrical and Computer Engineering, University of Tehran, Tehran, Iran

**Keywords:** deep learning, autism, children, diagnosis, facial image analysis

## Abstract

In this paper, we introduce a deep learning model to classify children as either healthy or potentially having autism with 94.6% accuracy using Deep Learning. Patients with autism struggle with social skills, repetitive behaviors, and communication, both verbal and non-verbal. Although the disease is considered to be genetic, the highest rates of accurate diagnosis occur when the child is tested on behavioral characteristics and facial features. Patients have a common pattern of distinct facial deformities, allowing researchers to analyze only an image of the child to determine if the child has the disease. While there are other techniques and models used for facial analysis and autism classification on their own, our proposal bridges these two ideas allowing classification in a cheaper, more efficient method. Our deep learning model uses MobileNet and two dense layers to perform feature extraction and image classification. The model is trained and tested using 3,014 images, evenly split between children with autism and children without it; 90% of the data is used for training and 10% is used for testing. Based on our accuracy, we propose that the diagnosis of autism can be done effectively using only a picture. Additionally, there may be other diseases that are similarly diagnosable.

## Introduction

### Motivation

Autism is primarily a genetic disorder, though there are some environmental factors, that cause challenges with social skills, repetitive behaviors, speech, and non-verbal communication (Alexander et al., 2007). In 2018, the Centers for Disease Control and Prevention (CDC) claimed that about 1 in 59 children will be diagnosed with some form of autism. Because there are so many forms of autism, it is technically called autism spectrum disorder (ASD) (Austimspeaks, 2019). A child can be diagnosed with ASD as early as 18 months old. Interestingly, while ASD is believed to be a genetic disorder, it is mainly diagnosed through behavioral attributes: “the ways in which children diagnosed with ASD think, learn, and problem-solve can range from highly skilled to severely challenged.” Early detection and diagnosis are crucial for any patient with ASD as this may significantly help them with their disorder.

We believe that facial recognition is the best possible way to diagnose a patient because of their distinct attributes. Scientists at the University of Missouri found that children diagnosed with autism share common facial feature distinctions from children who are not diagnosed with the disease (Aldridge et al., 2011; CBS News, 2017). The study found that children with autism have an unusually broad upper face, including wide-set eyes. They also have a shorter middle region of the face, including the cheeks and nose. Figure 1 shows some of these differences. Because of this, conducting facial recognition binary classification on images of children with autism and children who are labeled as healthy could allow us to diagnose the disease earlier and in a cheaper way.

**Figure 1:** On the **(Left)** is a child with autism, and on the **(Right)** is a child without autism, in order to compare some facial features.

### Data

In this work, we have used a dataset found on Kaggle, which consists of over three thousand images of both children with and without autism. This dataset is slightly unusual, as the publisher only had access to websites to gather all the images. When downloaded, the data is provided in two ways: split into training, testing, and validation vs. consolidated. If we decide to create our own machine learning model, the provided split of training, testing, and validating subgroups will be useful. The validation component will be important for determining the quality of the model we use, which means we do not have to strictly rely on the accuracy of the model to determine its quality. The training, testing, and validation subcategories are further split into autistic and non-autistic folders. The autistic training group consists of 1,327 images of facial images, and the non-autistic training directory consists of the same number of images. The autistic and non-autistic testing directories both have 140 images, for a total of 280 images. Lastly, the validation category has a total of 80 images: 40 facial images without autism and 40 with. If we can use a model already available, then using the consolidated images would be best, because that will allow us to control the amount used for training and testing (Gerry, 2020).

## State-of-the-Art

There have been several studies conducted using neural networks for facial, behavioral, and speech analysis (Eni et al., 2020; Liang et al., 2021). Most of these studies have focused on determining the age and gender of the individual in question (Iga et al., 2003). Additionally, there have been a few studies done focusing on the classification of autism using brain imaging modalities. Our work has taken the techniques available for facial analysis and applied these to the classification of autism.

### Facial Analysis

Wen-Bing Horng and associates (Horng et al., 2001) worked to classify facial images into one of four categories: babies, young adults, middle-aged adults, and old adults. Their study used two back-propagation neural networks for classification. The first focuses on geometric features, while the second focuses on wrinkle features. Their study achieved a 90.52% identification rate for the training images and 81.58% for the test images, which they noted is similar to a human's subjective justification for the same set of images. One of the complications noted by the researchers, which likely contributed to their seemingly low rates of success in comparison with other classification studies, was the fact that the age cutoffs for varying levels of “adults” do not typically have hard divisions, but for the sake of the study, this is necessary. For example, the researchers established the cutoff between young and middle adults at 39 years old (≤ 39 for young, >39 for middle). This creates issues when individuals are right at the boundary of two age groups. To prevent similar issues with our experiment, we decided to simply classify the images as “Autistic” and “Non-Autistic” rather than trying to additionally classify the levels of autism.

In a study by Shan (2012), researchers used Local Binary Patterns (LBP) to describe faces. Through the application of support vector machines (SVM), they were able to achieve a 94.81% success rate in determining the gender of the subject. The main breakthrough of this study was its ability to use only real-life images in their classification. Up to this point, many of the proven studies used ideal images, most of which were frontal, occlusion-free, with a clean background, consistent lighting, and limited facial expressions. Similar to this study, our facial images are derived from real-life environments and the dataset was constructed organically.

### Classification of Autism

A study conducted by El-Baz et al. (2007) focused on analyzing images of cerebral white matter (CWM) in individuals with autism to determine if classification could be achieved based only on the analysis of brain images. The CWM is first segmented from the proton density MRI and then the CWM gyrification is extracted and quantified. This approach used the cumulative distribution function of the distance map of the CWM gyrification to distinguish between the two classes: autistic and normal. While this study did yield successful results, the images were only taken from deceased individuals, so its success rate in classifying living individuals is still unknown. Our proposed classification system can achieve similar levels of accuracy (94.64%) while using significantly more subjects and only requiring an image of the individual rather than intensive, costly, brain scans, and subsequent detailed analysis.

### MobileNet

There are many different convolutional neural networks (CNN) available for image analysis (Hosseini, 2018; Hosseini et al., 2020b). Some of the more well-known models include GoogleNet, VGG-16, SqueezeNet, and AlexNet. Each of these distinct models offers different advantages, but MobileNet has been proven to be similarly effective while greatly reducing computation time and costs. MobileNet has shown that making their models thinner and wider has resulted in similar accuracy while greatly reducing multi-adds and parameters required for analysis (Tables 1–**3**).

**Table 1:** Depthwise separable vs. full convolution MobileNet (Jeatrakul and Wong, 2009; Howard et al., 2017).

**Model**	**ImageNet accuracy %**	**Million mult-adds**	**Million parameters**
Conv. MobileNet	71.7	4,866	29.3
MobileNet	70.6	569	4.2

In comparison with the previously mentioned models, MobileNet has been shown to be just as accurate while significantly reducing the computing power necessary to run the model (Tables 2, 3). Using this knowledge, we have decided that MobileNet is a sufficient model to use for our analysis.

**Table 2:** Narrow vs. shallow MobileNet and MobileNet width multiplier (Jeatrakul and Wong, 2009; Howard et al., 2017; Hosseini et al., 2020a).

**Model**	**ImageNet accuracy %**	**Million mult-adds**	**Million parameters**
Shallow MobileNet	65.3	307	2.9
1.0 MobileNet-224	70.6	569	4.2
0.75 MobileNet	68.4	325	2.6
0.5 MobileNet-224	63.7	149	1.3
0.25 MobileNet-224	50.6	41	0.5

**Table 3:** MobileNet resolution and MobileNet comparison to popular models.

**Model**	**ImageNet accuracy %**	**Million mult-adds**	**Million parameters**
1.0 MobileNet-224	70.6	569	4.2
1.0 MobileNet-192	69.1	418	4.2
1.0 MobileNet-160	67.2	290	4.2
1.0 MobileNet-128	64.4	186	4.2
GoogleNet	69.8	1,550	6.8
VGG 16	71.5	15,300	138

## Methods

In previous studies, children with autism have been found to have unusually wide faces and wide-set eyes. The cheeks and the nose are also shorter on their faces (Aldridge et al., 2011). In this study, deep learning has been used to train and learn about autism from facial analyses of children based on features that make them stand out from other children.

Our data set was obtained from Kaggle and consists of 3,014 children's facial images. Of these images, 1,507 images are presumed to have autism, and the remaining 1,507 are presumed to be healthy. Figure 2 shows a sample of images used for the training step. Images were obtained online, both through Facebook groups and through Google Image searches. Independent research was not conducted to determine if the individual in a picture was truly healthy or autistic. Once all the images were gathered, they were subsequently cropped so that the faces occupied most of the image. Before training, the images were split into three categories: train, validation, and test (Table 4). Images that were placed into each category must be put there manually. Therefore, repeatedly running the algorithm will generally produce the same results, assuming that the neural network ends up with the same weights. It is also worth noting that, currently, the global dataset has multiple repetitions, some of which are shared between the training, test, and validation datasets (Faris et al., 2016; Hosseini et al., 2017). It is, therefore, essential that these duplicates be cleaned out of the datasets before running the algorithm. For this case study, the duplicates have not yet been removed, which is likely improving overall accuracy.

**Figure 2:** Some images used in the deep learning training step. **(Top)** Children who have autism. **(Bottom)** Children who do not have autism.

**Table 4:** Dataset breakdown.

**Data set**	**Composition**	**Overall data composition %**
Train	1,327 autistic 1,327 healthy	88
Validation	80 autistic 80 healthy	5.3
Test	140 autistic 140 healthy	9.3
Total	1,507 autistic 1,507 healthy	100

Deep learning is broken down into three subcategories: CNN, pretrained unsupervised networks, and recurrent and recursive networks (Hosseini et al., 2016b). For this data set, we decided to use a CNN model. CNN can intake an image, assign importance to various objects within the image, and then differentiate objects within the image from one another. Additionally, CNNs are advantageous because the preprocessing involved is minimal compared to other methods. In this case, the input is the many images from the dataset to give an output variable: autistic or non-autistic. When looking at CNN, there are various kinds of methods to apply: LeNet, GoogLeNet, AlexNet, VGGNet, ResNet, and so forth. When trying to decide which CNN to use, it is crucial to consider what kind of data is in use, and the size of data being applied. For this instance, MobileNet is used because of the dataset: MobileNet is able to compute outputs much faster, as it can reduce computation and model size.

To perform deep learning on the dataset, MobileNet was utilized followed by two dense layers as shown in Figure 3. The first layer is dedicated to the distribution and allows customization of weights to input into the second dense layer. Thus, the second dense layer allows for classification. The architecture of MobileNet can be reviewed in Table 5.

**Figure 3:** The algorithm architecture of the proposed model, illustrating the use of MobileNet, followed by two dense layers to perform image recognition. MobileNet uses CNN to predict what is the shape of the object present and what is matched with it from the images.

**Table 5:** Body architecture of the developed MobileNet (Howard et al., 2017) for autism image recognition.

**Input size**	**Filter**	**Layer**	**Stride**
224 * 224 * 3	3 * 3 * 3 * 32	Convolution	S2
112 * 112 * 32	Depth-Wise 3 * 3 * 32	Depth-Wise Convolution	S1
112 * 112 * 32	1 * 1 * 32 * 64	Convolution	S1
112 * 112 * 64	Depth-Wise 3 * 3 * 64	Depth-Wise Convolution	S2
56 * 56 * 64	1 * 1 * 64 * 128	Convolution	S1
56 * 56 * 128	Depth-Wise 3 * 3 * 128	Depth-Wise Convolution	S1
56 * 56 * 128	1 * 1 * 128 * 128	Convolution	S1
56 * 56 * 128	Depth-wise 3 * 3 * 128	Depth-Wise Convolution	S2
28 * 28 * 128	1 * 1 * 128 * 256	Convolution	S1
28 * 28 * 256	Depth-Wise 3 * 3 * 256	Depth-Wise Convolution	S1
28 * 28 * 256	1 * 1 * 256 * 256	Convolution	S1
28 * 28 * 256	Depth-Wise 3 * 3 * 256	Depth-Wise Convolution	S2
14 * 14 * 256	1 * 1 * 256 * 512	Convolution	S1
14 * 14 * 512	Depth-Wise 3 * 3 * 512	Depth-Wise Convolution	S1
14 * 14 * 512	1 * 1 * 512 * 512	Convolution	S1
14 * 14 * 512	Depth-Wise 3 * 3 * 512	Depth-Wise Convolution	S1
14 * 14 * 512	1 * 1 * 512 * 512	Convolution	S1
14 * 14 * 512	Depth-Wise 3 * 3 * 512	Depth-Wise Convolution	S1
14 * 14 * 512	1 * 1 * 512 * 512	Convolution	S1
14 * 14 * 512	Depth-Wise 3 * 3 * 512	Depth-Wise Convolution	S1
14 * 14 * 512	1 * 1 * 512 * 512	Convolution	S1
14 * 14 * 512	Depth-Wise 3 * 3 * 512	Depth-Wise Convolution	S1
14 * 14 * 512	1 * 1 * 512 * 512	Convolution	S1
14 * 14 * 512	Depth-Wise 3 * 3 * 512	Depth-Wise Convolution	S2
7 * 7 * 512	1 * 1 * 512 * 1,024	Convolution	S1
7 * 7 * 1,024	Depth-Wise 3 * 3 * 1,024	Depth-Wise Convolution	S2
7 * 7 * 1,024	Depth-Wise 1 * 1 * 1,024	Convolution	S1
7 * 7 * 1,024	Pool 7 * 7	Average pooling	S1
1 * 1 * 1,024	1,024 * 1,000	Fully connected	S1
1 * 1 * 1,000	Classifier	Softmax	S1

For our MobileNet, an alpha of 1 and depth multiplier of 1 were utilized, thus we use the most baseline version of MobileNet. To make binary predictions from MobileNet, two fully connected layers are appended to the end of the model. The first is a dense layer with 128 neurons (L2 regularization = 0.015, ReLu activation) which is then connected to the prediction layer which only has two outputs (softmax activation). A dropout of 0.4 is applied to the first layer to prevent overfitting. The final output is a binary classification of either “autistic” or “non-autistic.”

The algorithm was run on an ASUS laptop (Beitou District, Taipei, Taiwan) with an Intel Core i7-6700HQ CPU at 2.60 GHz and 12 GB of RAM. The data was broken into batch sizes of 80. Upon completion of training and initial testing, the user can request additional training epochs.

## Results

The training was completed after ~15 epochs, yielding a test accuracy of 94.64%. Figure 4 shows how the loss of the training and test set changed with the continual addition of one epoch at a time. Figure 5 shows how accuracy (Hosseini et al., 2016a) changed for training, validation, and testing data with the continual addition of one epoch.

**Figure 4:** By adding one epoch at a time, this figure shows how the loss changes.

**Figure 5:** With the addition of one epoch, this figure shows how accuracy changed for training, validation, and testing data.

During the training, the weights that gave the validation set the highest accuracy were always stored. Therefore, if the accuracy decreased during a training set, there would be no ultimate loss of accuracy on the test set (Figures 1, 2). Similarly, if accuracy on the validation set decreased, the learning rate would also decrease during the next training session. Each epoch required ~10 min to run.

These preliminary results are very promising. Currently, there are many issues with the dataset that was used including duplicate images, improper age ranges, and lack of validation about the conditions of the individuals in each photo. Improving the data set could result in better results.

## Conclusion

While the statistics on how many children are diagnosed with autism are somewhat low, it is extremely important to diagnose as early as possible to provide the correct care for the patient. Additionally, the statistics on diagnosed children may be low because the method to accurately diagnose a child is somewhat ineffective. Thus, our classifier could prove to be very useful in diagnosing more children. Our results show that we have successfully achieved a high accuracy of 94.64%, meaning that it was able to identify a child with or without autism correctly about 95% of the time. To improve accuracy, cleaning the dataset would certainly help. Duplicates may falsely increase our test accuracy if an image is also in the training category. With more information about the individuals in the pictures, we could also ensure that age distributions are similar between the two populations. Currently, autism is rarely diagnosed in young children, so we would also ensure that no pictures of young children are in our dataset. Similarly, we could ensure that each category is “pure,” preventing false positives and false negatives. With these improvements, we would hope to get an accuracy >95%.

The success of this algorithm may also imply that other diseases can be diagnosed using only a picture, saving valuable time and resources in diagnosing other diseases and conditions. Down's Syndrome, for example, is another disease that markedly alters the facial features of those it afflicts. It is possible that, given sufficient and good data, our algorithm could distinguish between individuals with the disease and individuals without it.

## Data Availability Statement

Publicly available datasets were analyzed in this study. This data can be found at: https://www.kaggle.com/cihan063/autism-image-data.

## Author Contributions

M-PH defined and lead the project and defined the model and structures. MB, AH, and RM worked on the model. HS-Z proofread and organized the study for publication. All authors approved the final version of the manuscript for submission.

## Conflict of Interest

The authors declare that the research was conducted in the absence of any commercial or financial relationships that could be construed as a potential conflict of interest.

## Publisher's Note

All claims expressed in this article are solely those of the authors and do not necessarily represent those of their affiliated organizations, or those of the publisher, the editors and the reviewers. Any product that may be evaluated in this article, or claim that may be made by its manufacturer, is not guaranteed or endorsed by the publisher.

## References

[B1] AldridgeK.GeorgeI. D.ColeK. K.AustinJ. R.TakahashiT. N.DuanY.. (2011). Facial phenotypes in subgroups of prepubertal boys with autism spectrum disorders are correlated with clinical phenotypes. Mol. Autism 2, 1–12. 10.1186/2040-2392-2-1521999758PMC3212884

[B2] AlexanderA. L.LeeJ. E.LazarM.BoudosR.DuBrayM. B.OakesT. R.. (2007). Diffusion tensor imaging of the corpus callosum in autism. Neuroimage 34, 61–73. 10.1016/j.neuroimage.2006.08.03217023185

[B3] Austimspeaks (2019). What Is Autism? Austimspeaks. Available online at: https://www.autismspeaks.org/what-autism (accessed March 11, 2020).

[B4] CBS News (2017). Is it Autism? Facial Features That Show Disorder. CBS News. Available online at: https://www.cbsnews.com/pictures/is-it-autism-facial-features-that-show-disorder/8/ (accessed March 12, 2020).

[B5] El-BazA.CasanovaM. F.Gimel'farbG.MottM.SwitwalaA. E. (2007). A new image analysis approach for automatic classification of autistic brains, in 2007 4th IEEE International Symposium on Biomedical Imaging: From Nano to Macro (Arlington, VA: IEEE), 352–355. 10.1109/ISBI.2007.356861

[B6] EniM.DinsteinI.IlanM.MenasheI.MeiriG.ZigelY. (2020). Estimating autism severity in young children from speech signals using a deep neural network. IEEE Access 8, 139489–139500. 10.1109/ACCESS.2020.301253227295638

[B7] FarisH.AljarahI.MirjaliliS. (2016). Training feedforward neural networks using multi-verse optimizer for binary classification problems. Appl. Intell. 45, 322–332. 10.1007/s10489-016-0767-1

[B8] Gerry (2020). Autistic Children Data Set. Kaggle.

[B9] HorngW. B.LeeC. P.ChenC. W. (2001). Classification of age groups based on facial features. Tamkang Instit. Technol. 4, 183–192. 10.6180/jase.2001.4.3.05

[B10] HosseiniM. P. (2018). Brain-Computer Interface for Analyzing Epileptic Big Data. (Doctoral dissertation), New Brunswick, NJ: Rutgers University-School of Graduate Studies.

[B11] HosseiniM. P.HosseiniA.AhiK. (2020a). A Review on machine learning for EEG Signal processing in bioengineering. IEEE Rev. Biomed. Eng. 14, 204–218. 10.1109/RBME.2020.296991532011262

[B12] HosseiniM. P.LuS.KamarajK.SlowikowskiA.VenkateshH. C. (2020b). Deep learning architectures, in Deep Learning: Concepts and Architectures (Cham: Springer), 1–24. 10.1007/978-3-030-31756-0_1

[B13] HosseiniM. P.Nazem-ZadehM. R.PompiliD.Jafari-KhouzaniK.ElisevichK.Soltanian-ZadehH. (2016a). Comparative performance evaluation of automated segmentation methods of hippocampus from magnetic resonance images of temporal lobe epilepsy patients. Med. Phys. 43, 538–553. 10.1118/1.493841126745947PMC4706546

[B14] HosseiniM. P.PompiliD.ElisevichK.Soltanian-ZadehH. (2017). Optimized deep learning for EEG big data and seizure prediction BCI via internet of things. IEEE Trans. Big Data 3, 392–404. 10.1109/TBDATA.2017.276967027295638

[B15] HosseiniM. P.Soltanian-ZadehH.ElisevichK.PompiliD. (2016b). Cloud-based deep learning of big EEG data for epileptic seizure prediction, in 2016 IEEE Global Conference on Signal and Information Processing (GlobalSIP) (Washington, DC: IEEE), 1151–1155. 10.1109/GlobalSIP.2016.7906022

[B16] HowardA. G.ZhuM.ChenB.KalenichenkoD.WangW.WeyandT.. (2017). Mobilenets: Efficient convolutional neural networks for mobile vision applications. arXiv [Preprint] arXiv:1704.04861.

[B17] IgaR.IzumiK.HayashiH.FukanoG.OhtaniT. (2003). A gender and age estimation system from face images, in SICE 2003 Annual Conference (IEEE Cat. No. 03TH8734), Vol. 1 (Fukui: IEEE), 756–761.

[B18] JeatrakulP.WongK. W. (2009). Comparing the performance of different neural networks for binary classification problems, in 2009 Eighth International Symposium on Natural Language Processing (Bangkok: IEEE), 111–115. 10.1109/SNLP.2009.5340935

[B19] LiangS.SabriA. Q. M.AlnajjarF.LooC. K. (2021). Autism spectrum self-stimulatory behaviors classification using explainable temporal coherency deep features and SVM classifier. IEEE Access 9, 34264–34275. 10.1109/ACCESS.2021.3061455

[B20] ShanC. (2012). Learning local binary patterns for gender classification on real-world face images. Patt. Recogn. Lett. 33, 431–437. 10.1016/j.patrec.2011.05.016

